The article "Preparation of Porous Ceramic Building Decoration Materials by Foaming Method and Research on Nanomechanical Properties" was retracted in 2023. Reasons: signs of a paper mill; compromised peer review; unreliable results or conclusions.

# Preparation of Porous Ceramic Building Decoration Materials by Foaming Method and Research on Nanomechanical Properties

**DOI:** 10.1155/2022/8339503

**Published:** 2022-05-14

**Authors:** Hongyao Zhang

**Affiliations:** Shazhou Professional Institute of Technology, Zhangjiagang, Jiangsu 215600, China

## Abstract

Because of its excellent properties, mullite porous ceramics are widely used in thermal insulation materials, catalyst carriers, gas-liquid filtration, separation materials, etc. At the same time, zirconia not only has the advantages of high melting point, good chemical stability, and high strength but also can significantly improve the strength of ceramics through phase transformation and particle dispersion in the matrix and is widely used in the reinforcement of ceramics. In this paper, using mullite powder as the raw material, Al_2_O_3_ and SiO_2_/ZrSiO_4_ as the starting material for the mullite self-bonding phase, and AlF_3_·3H_2_O, ZrO_2,_ and Y_2_O_3_ as additives, the zirconia-reinforced mullite was prepared by the foaming-injection method. The volume density, linear shrinkage rate, microstructure, room temperature, etc. of nanozirconia-reinforced mullite porous ceramics were studied by the amount of the foaming agent, the amount of mullite self-bonding phase powder, the type and amount of additives, etc. Effects of mechanical properties and thermal conductivity were also analyzed. The research results show that zirconia-reinforced mullite porous ceramics were prepared with mullite powder and 6 wt% AlF_3_·3H_2_O as raw materials, and ZrO_2_ and Y_2_O_3_ as additives. Adding an appropriate amount of ZrO_2_ and Y_2_O_3_ can significantly improve the mechanical properties of porous ceramics. When ZrO_2_ is 6 wt% and Y_2_O_3_ is 8 wt%, the porosity is 66.4% and the flexural strength and compressive strength of porous ceramics with a large pore size of 168 *μ*m can reach 14.3 MPa and 36.3 MPa, respectively, which are obviously better than the strength of mullite porous ceramics without adding Y_2_O_3_ (flexural strength 11.3 MPa, nanocompressive strength 29.4 MPa).

## 1. Introduction

Porous ceramics refer to porous ceramic materials with open and closed pore diameters and high porosity fired at high temperatures. They not only have large porosity, high specific surface area, and low density but also have the advantages of low thermal conductivity, and have excellent properties such as energy absorption, damping characteristics, and uniform gas-liquid permeability [1–3]. It is often widely used as melt, gas and solid filters, catalyst carriers, electrolytic membranes, high-pressure gas and sound wave-absorbing materials, thermal insulation materials, biomedical materials, etc. [4–6].

The article "Preparation of Porous Ceramic Building Decoration Materials by Foaming Method and Research on Nanomechanical Properties" was retracted in 2023. Reasons: signs of a paper mill; compromised peer review; unreliable results or conclusions.

Mullite porous ceramics are widely used in energy recovery, metal smelting industry, and chemical industry due to their high melting point, good acid and alkali corrosion resistance, high porosity, good mechanical properties, high temperature resistance, low thermal conductivity, and other excellent properties. They are also used in the pharmaceutical industry, biomedical industry, military industry, and other fields. The preparation methods of mullite porous ceramics mainly include the foaming-injection molding method, organic foam impregnation method, adding pore-forming agent method, freeze-drying method, sol-gel method, biological template method, and ion exchange method. Among them, the foam-injection molding method has become one of the research hotspots in recent years because of its simple process and the ability to prepare large-sized and complex products. However, the traditional foaming-injection molding method needs to add a large amount of organic matter when preparing porous ceramics. During the sintering process, the organic matter decomposes and volatilizes a large amount of harmful gases, causing environmental pollution and seriously affecting the mechanical properties of porous ceramics. At the same time, the porous ceramic prepared by the traditional foaming method has a large shrinkage rate, and microcracks will form on the surface of the sample, thereby reducing the mechanical properties of the porous ceramic. It is difficult to prepare mullite porous ceramics with high porosity, high strength, and low shrinkage rate. Therefore, how to improve the porosity and mechanical properties of mullite porous ceramics by improving the process is a new research direction in the future. The process of preparing a porous foam glass-ceramic composite building thermal insulation material by a foaming method is shown in Figure 1.

In this paper, the foaming-injection molding combined with the reaction sintering method is proposed to prepare zirconia-reinforced mullite porous ceramics with high porosity, high strength, and low thermal conductivity by introducing the zirconia-reinforcing phase, additives, and self-bonding phase. Its phase composition, linear shrinkage, bulk density, porosity, microstructure, pore size, mechanical properties, and thermal conductivity were studied.

## 2. Literature Review

The organic foam impregnation method [7–9] is a widely used method for preparing porous lightweight ceramics in the industry. This method was first proposed by Zhang et al. [10] in 1963. The main process is to fully immerse the organic foam with a three-dimensional network structure into the prepared ceramic slurry, then remove the excess slurry on the surface of the foam board, and finally obtain porous ceramics after drying and sintering.

The article "Preparation of Porous Ceramic Building Decoration Materials by Foaming Method and Research on Nanomechanical Properties" was retracted in 2023. Reasons: signs of a paper mill; compromised peer review; unreliable results or conclusions.

Czelusniak and Amorim. [11] used *α*-Al_2_O_3_ as raw material, gum arabic as dispersant, and organic foams with different pore sizes as templates. After sintering at 1200°C/2 h by the organic foam impregnation method, porous alumina with a porosity of up to 93% was prepared. The effects of dispersant and sintering aid dosage, sintering temperature, and other factors on the properties of porous ceramics were mainly studied. Teng et al. [12] used Ti_2_AlN powder as raw material, polyacrylamide as the dispersant, polyvinyl alcohol as the binder, and ethanol as a defoamer, treated the polyurethane sponge with NaOH solution, and soaked it with hydroxymethyl cellulose solution. Ti_2_AlN porous ceramics with a three-dimensional framework structure and relatively uniform pores were prepared. Zhou et al. [13] used ZrO_2_ as the raw material, MgO and CeO_2_ as stabilizers, and prepared ZrO_2_ porous ceramics with an excellent performance by sintering organic foam impregnation method. The effects of stabilizer types on shrinkage, surface morphology, and high-temperature phase content of ceramic samples were studied. The results show that using CeO_2_ as a stabilizer can reduce the linear shrinkage of the sample, and using a composite stabilizer of MgO and CeO_2_ to promote sintering and generate a high-temperature stable phase is beneficial to improve the sintering rate of the sample.

Although the above research can prepare porous ceramics with excellent properties, there are still some problems with this method: (1) the affinity of the organic foam template with the ceramic slurry affects the thickness and uniformity of the slurry coverage; (2) the body is easily deformed during the sintering process, and the pores of the hollow structure formed by the organic matter after burning have a great influence on the strength of the porous ceramic product; (3) the organic foam emits a large amount of harmful gases during sintering, pollutes the environment, and is harmful to human health; (4) the pore size and porosity of the prepared porous ceramics are limited by the shape and pore size of the selected organic foam template, and the requirements for the pore size of the template are relatively strict. In order to improve the pore size distribution and mechanical properties, many scholars generally use methods combined with freeze-drying, adding pore-forming agents, etc. to prepare porous ceramics.

The foaming method is to add a certain proportion of organic substances such as water-reducing agent, binder, or dispersant to the prepared ceramic slurry, and generate a large number of bubbles through a chemical reaction, mechanical foaming, etc., and then natural drying combined with hot air drying, after sintering at a specific temperature to obtain porous ceramic products [14–16]. The preparation process is shown in Figure 2. During the experiment, some organic substances are often used as a foaming agent, water-reducing agent, binder, dispersing agent, etc. There are many types of commonly used foaming agents, which are mainly divided into physical foaming agents and chemical foaming agents. Physical foaming agents include liquid carbon dioxide, cyclopentane, hydrofluoroalkane, n-hexane, petroleum ether, dichlorodifluoromethane, hydrogenated polyether, etc. Chemical foaming agents include N-diterephthalidene (NTA), azobisisobutyronitrile, diethyl azodicarboxylate, 4-disulfonylhydrazide diphenyl ether, etc. Superplasticizers and dispersants generally include lignosulfonate sodium salt superplasticizers, naphthalene-based superplasticizers, amino superplasticizers, aliphatic superplasticizers, polycarboxylate superplasticizers, and the like. Adhesives mainly include instant-drying, anaerobic, pressure-sensitive, hot-melt, thermosetting, etc. [17].

The article "Preparation of Porous Ceramic Building Decoration Materials by Foaming Method and Research on Nanomechanical Properties" was retracted in 2023. Reasons: signs of a paper mill; compromised peer review; unreliable results or conclusions.

Mullite porous ceramics are widely used in various fields due to their many advantages. However, by reviewing and summarizing the research on mullite porous ceramics in recent years, it is found that there are still some urgent problems to be solved in the preparation method and performance of mullite porous ceramics, which are also common problems of various types of porous ceramics [18]. For example, (1) the shrinkage rate of mullite porous ceramics is relatively large during the sintering process; (2) a large amount of organic matter is added during the preparation process, and harmful gases are released during sintering to pollute the environment and human health; (3) the preparation methods of ceramics all have their disadvantages more or less; (4) the prepared mullite porous ceramics have low mechanical strength due to high brittleness, cracking, and other reasons. In view of the above problems, this paper intends to prepare zirconia-reinforced mullite porous ceramics by foaming-injection combined with an in-situ reaction sintering method so as to provide a reference for the performance improvement of porous ceramics and a guarantee for environmental protection.

## 3. Experimental Method

### 3.1. Experimental Materials and Equipment

The raw materials and specifications used in the experiment are shown in Table 1:

Table 2 shows the particle size characteristic parameters of the experimental raw materials before and after ball milling. It can be seen from the table that the average particle size (Dav) of ZrO_2_ powder decreased from 49.8 *μ*m before ball milling to 9.1 *μ*m after ball milling for 4 hours, and the median particle size (D50) decreased from 45.9 *μ*m decreased to 7.2 *μ*m. While the specific surface area (S/V) increased from 0.1 m^2^/cm^3^ to 0.7 m^2^/cm^3^, the particle size before ball milling was mainly distributed between 24∼80 *μ*m, and the particle size distribution after ball milling was mainly between 2 and 20 *μ*m. It can be seen from the above that ball milling can effectively reduce the particle size of ZrO_2_ powder; for ZrSiO_4_ powder before and after ball milling, the average particle size, median particle size, and specific surface area change very little, and the particle size after ball milling is very small. It is mainly distributed between 0.3 and 1.4 *μ*m; the particle size of composite powder after ball milling is mainly distributed between 0.4 and 1.4 *μ*m.

The article "Preparation of Porous Ceramic Building Decoration Materials by Foaming Method and Research on Nanomechanical Properties" was retracted in 2023. Reasons: signs of a paper mill; compromised peer review; unreliable results or conclusions.

### 3.2. Experimental Procedure

First, according to the mass ratio of corundum ball : powder : water of 10 : 5 : 3, a certain amount of corundum ball was weighed, mixed the powder (zirconium silicate, alumina, and aluminum fluoride or yttrium oxide in a certain proportion), deionized water, put it into a ball milling tank, ball-milled on a planetary ball mill at a speed of 250 r/min for 4 hours, put the obtained ceramic slurry in a blast drying oven at 120°C to dry to constant weight, passed through a 100-mesh sieve, and obtained a mixed powder body.

Then, the solid content of the mixed powder was controlled to be 52 vol%, a certain amount of the mixed powder was weighed and gradually added to the aqueous solution containing 0.4 wt% Isobam104 (IB, relative to the mass of the powder), and the pulp with good fluidity is obtained after rapid stirring.

Then, a certain amount of lauryl sulfate triethanolamine (0.2∼1 vol%, relative to the volume of the slurry) foaming agent was added into the slurry, firstly through high-speed mechanical stirring and then low-speed stirring to foam to obtain a foam slurry with uniform bubbles. Then,it was quickly injected into a 220 mm × 160 mm × 40 mm mold to solidify and form, the poured mold was let to stand at room temperature for 24 h to demold, and first dried the green body in the natural environment for 72 h, and then heated it at 40∼110°C. Then, it was dried in a drying oven until all moisture evaporates.

Finally, the dried green body was placed in an alumina crucible, slowly put into a box-type sintering furnace (specification KSS-1700°C) in an air atmosphere, heated to 1600°C at 3°C/min and kept for 2 h, and cooled with the furnace to 1600°C. The zirconia reinforced mullite porous ceramic is obtained after room temperature.

The article "Preparation of Porous Ceramic Building Decoration Materials by Foaming Method and Research on Nanomechanical Properties" was retracted in 2023. Reasons: signs of a paper mill; compromised peer review; unreliable results or conclusions.

### 3.3. Specimen Performance Testing and Characterization

The bulk density of porous ceramics can be directly calculated from the mass-to-volume ratio of the sintered sample [19].

The porosity of porous ceramics can be measured by the Archimedes method. First, the samples are dried in a blast drying oven at 100°C ± 5°C, then cooled to room temperature in the drying oven, and then weighed to obtain dryness. The mass of the sample is 1 m. The sample was put into a clean beaker, placed in a vacuum desiccator, evacuated until the residual pressure is less than 10 mmHg, keep it for 10 min, then opened the valve of the upper funnel of the vacuum desiccator, and let the tap water flow naturally until the sample is completely dry. When submerged but no bubbles are generated, the valve was closed.

The sample was taken out of the water, a moisture-absorbing cloth was used to dry the liquid on the outer surface of the wet sample, and then weighed the sample was quickly weighed to the nearest 0.01 g to obtain the wet sample mass *m*_2_.

Then, the mass (floating weight) of the sample was measured in a suspended state in water, accurate to 0.01 g, to obtain a floating weight of 3 m. The absorbent cloth should be immersed in water in advance and completely soaked and wrung out gently to avoid absorbing the water in the pores of the ceramic sample and affecting the experimental results. It is calculated as follows:

(1) $$\begin{array}{c} \pi_{\alpha }=\frac{m_{2}-m_{1}}{m_{2}-m_{3}}\times 100\%. \end{array}$$

where *π*_*α*_ is the apparent porosity (%), *m*_1_ is the mass of the dry sample (g), *m*_2_ is the mass of the wet sample (g), and *m*_3_ is the floating weight (g).

The flexural strength is measured by the three-point bending method, which can be calculated according to the following formula (2), with a span of 100 mm. The size of the sample is 150 mm × 25 mm × 25 mm.

(2) $$\begin{array}{c} \sigma_{F}=\frac{3}{2}\times \frac{F_{\max}L_{s}}{bh^{2}}, \end{array}$$

where *σ*_*F*_ is the flexural strength at room temperature (MPa), *F*_max_ is the maximum pressure applied to the sample (N), *L*_*s*_ is the distance between the lower knife edges (mm), *b* is the width of the sample (mm), and *h* is the height of the sample (mm).

## 4. Result Analysis

In the reinforcement mechanism of mullite porous ceramics, the second phase of mullite porous ceramics is introduced for reinforcement. The reinforcement method is changed from single whisker reinforcement to phase particle composite reinforcement, whisker-particle composite reinforcement, and whisker-phase transition composite reinforcement, thereby improving the mechanical properties of mullite porous ceramics [20]. The enhancement of ZrO_2_, especially the enhancement of Y_2_O_3_-stabilized tetragonal phase ZrO_2_, makes the matrix show higher strength. Therefore, adding ZrO_2_ to the mullite matrix can be used to improve the mechanical properties of mullite and improve the mechanical strength. Liu et al. [21] used zirconium quartz and bauxite as raw materials, and added CaO, Y_2_O_3_, and MgO as additives, and prepared zirconia reinforced mullite ceramics with a compressive strength of up to 620 MPa by hot pressing sintering. Chen et al. [22] used mullite as raw material, coarse and fine ZrO_2_ (Y_2_O_3_) as admixtures, and prepared zirconia reinforced mullite ceramics with a compressive strength of 378 MPa by isostatic pressing. Hussien et al. [23] used fused mullite, *α*-Al_2_O_3_ micropowder and semistable zirconia as raw materials, polycrystalline alumina fiber as admixture, and sintered at 1500°C for 3 h to prepare a composite material with good dimensional stability and flexural strength. and compressive strength of 56 MPa and 203 MPa, respectively, and the number of thermal shocks up to 36 times of alumina fiber reinforced mullite-zirconia composite ceramics [24].

The article "Preparation of Porous Ceramic Building Decoration Materials by Foaming Method and Research on Nanomechanical Properties" was retracted in 2023. Reasons: signs of a paper mill; compromised peer review; unreliable results or conclusions.

In this paper, mullite and 6 wt% AlF_3_·3H_2_O were used as raw materials, ZrO_2_ was used as reinforcing phase, and Y_2_O_3_ additive was used to prepare zirconia reinforced mullite porous ceramics by foaming-injection method. Influence of mechanical properties of stone porous ceramic samples.

### 4.1. Effect of ZrO_2_ on Mechanical Properties of Mullite Porous Ceramics

When using different amounts of ZrO_2_, the XRD of the mullite porous ceramics prepared after sintering at 1550°C/2 h with the increase of the amount of ZrO_2_, the diffraction peaks of mullite did not change significantly, while the diffraction peaks of ZrO_2_ increased gradually. When ZrO_2_ is not added, there are only mullite phase and *α*-Al_2_O_3_ phase in the porous ceramic sample, and *α*-Al_2_O_3_ phase appears mainly due to the decomposition reaction of AlF_3_·3H_2_O. When the amount of ZrO_2_ is 3 wt%, the main crystal phase in the sample is mullite phase, and the secondary crystal phase is *α*-Al_2_O_3_ phase. At the same time, the diffraction peak of m-ZrO_2_ appears, and the intensity of the diffraction peak of m-ZrO_2_ continuously enhanced. It shows that the addition of ZrO_2_ has no obvious effect on the composition of mullite porous ceramics.

Figure 3 shows the effect of the amount of ZrO_2_ on the flexural strength and compressive strength of the mullite porous ceramics prepared by sintering at 1550°C/2 h. It can be seen that the flexural strength and compressive strength of porous ceramics increase with the increase of the amount of ZrO_2_. When the amount of zirconia was 9 wt%, the flexural strength and compressive strength of the prepared porous ceramic samples were 12.6 MPa and 33.7 MPa, respectively, which were 25.4% and 23.7% higher than those of the samples without ZrO2 addition, respectively. This is mainly due to the addition of ZrO_2_, which reduces the pore size of porous ceramics, and the distribution of pores is more uniform, which is beneficial to improve its strength. In addition, ZrO_2_ particles are uniformly distributed in the mullite matrix. During the growth of mullite columnar crystals, the intense “pinning effect” of ZrO_2_ particles hinders the movement of grain boundaries and limits the growth of mullite columnar crystals (this is consistent with the high-magnification SEM picture), which plays the role of refining the particles. When the columnar crystal matrix encounters the ZrO_2_ particles, due to the “pinning effect,” the grain boundary will deflect and absorb a large amount of energy, and the mullite columnar crystals are staggered and densely arranged. The densification of grains and columnar crystals caused by the “pinning effect” of cloth and ZrO_2_ particles consumes a lot of fracture energy, thereby improving the mechanical properties of mullite porous ceramics.

The article "Preparation of Porous Ceramic Building Decoration Materials by Foaming Method and Research on Nanomechanical Properties" was retracted in 2023. Reasons: signs of a paper mill; compromised peer review; unreliable results or conclusions.

### 4.2. Effect of Y_2_O_3_ on Mechanical Properties of Mullite Porous Ceramics

Figure 4 shows the effect of the amount of wY_2_O_3_ on the flexural strength and compressive strength of the mullite porous ceramics prepared after sintering at 1550°C/2 h. It can be seen from this that the mechanical strength of porous ceramics increases with the increase of the amount of Y_2_O_3_. When the amount of Y_2_O_3_ was 8 wt%, the flexural strength and compressive strength of the prepared porous ceramics reached the maximum, which were 14.3 MPa and 36.3 MPa, respectively, which were 20.5% and 19% higher than the strengths of mullite porous ceramics with similar porosity prepared without additives. This is mainly due to the addition of Y_2_O_3_, which completely converts m-ZrO_2_ into t-ZrO_2_; on the other hand, combined with the high-magnification SEM image, it can be seen that with the increase of the amount of Y_2_O_3_, solid solution reaction occurs between particles, resulting in a eutectic. The particles continue to infiltrate between the particles, the particles are refined, and the grain boundaries of the ceramics gradually become smaller. Combining the above reasons, it is beneficial to improve the strength of mullite porous ceramics.

## 5. Conclusion

In this paper, zirconia-reinforced mullite porous ceramics were prepared by the foaming-injection molding method, and the bulk density, porosity, microstructure, mechanical properties, and thermal insulation properties of porous ceramics were studied. The main conclusions are as follows: zirconia-reinforced mullite porous ceramics were prepared using mullite and 6 wt% AlF_3_·3H_2_O as raw materials, and ZrO_2_ and Y_2_O_3_ as additives. Introducing an appropriate amount of ZrO_2_ and Y_2_O_3_ can significantly improve the mechanical properties of porous ceramics. When only 6 wt% ZrO_2_ is added, the flexural strength and compressive strength of the prepared zirconia reinforced mullite porous ceramics with a porosity of 68.6% are 11.3 MPa and 29.4 MPa, respectively. On this basis, when Y_2_O_3_ is added at 8 wt%, the porosity of the prepared porous ceramics is 66.4%, and the flexural strength and compressive strength of the porous ceramics with a large pore diameter of 168 *μ*m can reach 14.3 MPa and 36.3 MPa, respectively, which is higher than that of adding only 6 wt%. The flexural strength and compressive strength of ZrO_2_ porous ceramics are increased by 20.5% and 19%, respectively.

The article "Preparation of Porous Ceramic Building Decoration Materials by Foaming Method and Research on Nanomechanical Properties" was retracted in 2023. Reasons: signs of a paper mill; compromised peer review; unreliable results or conclusions.

In this paper, zirconia-reinforced mullite porous ceramics were prepared by the foaming-injection method, and their bulk density, porosity, linear shrinkage, mechanical properties at room temperature and thermal insulation properties were studied. However, due to the time, its high-temperature mechanical properties and high-temperature thermal insulation properties have not been studied [25]. In addition, the selection of types and amounts of additives is not comprehensive enough. It can be further improved in future research. The mechanical properties and thermal insulation properties of mullite porous ceramics can be further improved by improving the experimental scheme or sintering process.

## Figures and Tables

**Figure 1:** Schematic diagram of the preparation of porous foam glass-ceramic composite building thermal insulation material by the foaming method.

**Figure 2:** Process flow of preparing porous ceramics by the foaming method.

**Figure 3:** Effect of ZrO_2_ amount on flexural strength and compressive strength of mullite porous ceramics.

**Figure 4:** Effect of Y_2_O_3_ amount on flexural strength and compressive strength of mullite porous ceramics.

**Table 1:** Raw materials used in experiments.

Raw material name	Molecular formula	Purity	Origin
Zirconium silicate	ZrSiO_4_	Industrial grade	Shan Dong
Alumina	*α*-Al_2_	Industrial grade	Qing Dao
Mullite	3Al_2_O_3_·2SiO_2_	DM-70 (325 mesh)	Shan Dong
Silica	SiO_2_	≥99.2%	Qing Huang Dao
Yttrium oxide	Y_2_O_3_	Chemically pure (CP)	Shang Hai
Zirconia	ZrO_2_	≥99.80	Ping Xiang

The article "Preparation of Porous Ceramic Building Decoration Materials by Foaming Method and Research on Nanomechanical Properties" was retracted in 2023. Reasons: signs of a paper mill; compromised peer review; unreliable results or conclusions.

**Table 2:** Characteristic parameters of particle size distribution before and after ball milling of raw materials.

Characteristic parameters	D10 (*μ*m)	D50 (*μ*m)	D90 (*μ*m)	D97 (*μ*m)	Dav (*μ*m)	S/V (m^2^/cm^3^)	＜10 *μ*m (%)	＜20 *μ*m (%)
Before ZrO_2_ ball milling	23.2	45.9	81.2	1.7	49.8	0.1	0.5	6.7
After ZrO_2_ ball milling for 4 h	1.3	7.2	19.8	26.9	9.1	0.7	64.1	90.2
ZrSiO_4_ before ball milling	0.4	0.8	1.7	2.4	1.0	7.1	100	100
After ZrSiO_4_ ball milling for 4 h	0.3	0.6	1.3	1.7	0.7	9.1	100	100
ZrSiO_4_ and Al_2_O_3_ after ball milling for 4 h	0.3	0.7	1.3	1.7	0.7	9.1	100	100

## Data Availability

The data used to support the findings of this study are available from the corresponding author upon request.

## References

[1] Shi J., Chen Z., Zheng B. (2021). Experimental research on material and mechanical properties of rock-like filling materials in disaster prevention of underground engineering. *Advances in Materials Science and Engineering*.

[2] Sadasivan N., Balasubramanian M. (2021). Severe plastic deformation of tubular materials—process methodology and its influence on mechanical properties—a review. *Materials Today Proceedings*.

[3] Lucio M. D. S., Kultayeva S., Kim Y. W., Song I. H. (2021). Effects of sic whisker addition on mechanical, thermal, and permeability properties of porous silica-bonded sic ceramics. *International Journal of Applied Ceramic Technology*.

[4] Owaid A. A., Kaygusuz H., Mohammed F. M. (2021). Effect of reinforcing materials on mechanical properties of composite material using taguchi method. *Journal of Physics: Conference Series*.

[5] Yang Z., Xie Y., He J., Wang F., Zeng X., Ma K. (2021). A comparative study on the mechanical properties and microstructure of cement-based materials by direct electric curing and steam curing. *Materials*.

[6] Yang Z., Li K., Ma S., Yu J., Ren Z. (2021). Preparation, mechanical and leaching properties of cazro3 ceramic cores. *International Journal of Applied Ceramic Technology*.

[7] Liu D., Wang W., Zha X., Guo R., Jiao H. (2021). Effects of groove on the microstructure and mechanical properties of dissimilar steel welded joints by using high-entropy filler metals. *Journal of Materials Research and Technology*.

[8] Li X., Wu Y. J., Ding M. (2021). Research on the relationship between carbon precipitation and mechanical properties of dissimilar steel welds. *Journal of Physics: Conference Series*.

[9] Vattur Sundaram M., Hryha E., Chasoglou D., Rottstegge A., Nyborg L. (2022). Effect of density and processing conditions on oxide transformations and mechanical properties in Cr–Mo-alloyed pm steels. *Metallurgical and Materials Transactions A*.

The article "Preparation of Porous Ceramic Building Decoration Materials by Foaming Method and Research on Nanomechanical Properties" was retracted in 2023. Reasons: signs of a paper mill; compromised peer review; unreliable results or conclusions.

[10] Zhang W., Chen L., Xu C. (2021). Densification, microstructure and mechanical properties of multicomponent (tizrhfnbtamo) c ceramic prepared by pressureless sintering. *Journal of Materials Science & Technology*.

[11] Czelusniak T., Amorim F. L. (2021). Influence of energy density on polyamide 12 processed by sls: from physical and mechanical properties to microstructural and crystallization evolution. *Rapid Prototyping Journal*.

[12] Teng J., Liu P. Y., Li Z. H., Qi Y. H. (2021). *Mechanical Properties and Seismic Performance Research on Primary-Secondary Structure for High-Rise Building*.

[13] Zhou H., Li H., Mei Y., Wang G., Liu C. (2021). Research on vibration reduction method of nonpneumatic tire spoke based on the mechanical properties of domestic cat’s paw pads. *Applied Bionics and Biomechanics*.

[14] Kai X., Wu L., Peng Y. (2021). Effects of zr element on the microstructure and mechanical properties of b4c/al composites fabricated by melt stirring method. *Composites Part B: Engineering*.

[15] Wang J., Wang G., Zhao J., Zhang A., Dong G., Wang X. (2021). Research on cellular morphology and mechanical properties of microcellular injection–molded bcpp and its blends. *International Journal of Advanced Manufacturing Technology*.

[16] Sinković T., Jambreković B., Sedlar T. (2021). Interpreting research results for the physical and mechanical properties of wood: an approach not dependent on a juvenile/mature wood boundary. *Bioresources*.

[17] Gao X., Zhang Z., Huang X. (2021). Research on mesomechanical properties of rock and soil considering shape factors. *Hans Journal of Civil Engineering*.

[18] Gurumurthy O., Venkateswaran S. (2022). Experimental studies and regression analysis on mechanical properties of MMCs based zinc-aluminium alloys with graphite particles reinforcement. *Materials Today: Proceedings*.

[19] Jiang X., Chu F., Zhou X. (2022). Construction of bismaleimide resin with enhanced flame retardancy and mechanical properties based on a novel DOPO-derived bismaleimide monomer. *Journal odf Colloid and Interface Science*.

[20] Li X., Zhou Y., Guo Z. (2022). Influence of different substrates on the microstructure and mechanical properties of WC-12Co cemented carbide fabricated via laser melting deposition. *International Journal of Refracroty Metals and Hard Materials*.

[21] Liu W., Chen X., Ahmad T. (2022). Microstructures and mechanical properties of Cu–Ti alloys with ultrahigh strength and high ductility by thermo-mechanical treatment. *Materials Science and Engineering: A*.

[22] Chen B., Xiao G., Yi M., Zhang J., Zhou T., Chen Z. (2021). Mechanical properties and microstructure of al2o3/tib2 and al2o3/tib2/gnps ceramic tool materials prepared by spark plasma sintering. *Ceramics International*.

The article "Preparation of Porous Ceramic Building Decoration Materials by Foaming Method and Research on Nanomechanical Properties" was retracted in 2023. Reasons: signs of a paper mill; compromised peer review; unreliable results or conclusions.

[23] Hussien R. M., Abd el-Hafez L. M., Mohamed R. A. S., Faried A. S., fahmy N. G. (2021). Influence of nano waste materials on the mechanical properties, microstructure, and corrosion resistance of self-compacted concrete. *Case Studies in Construction Materials*.

[24] Bradha M., Balakrishnan N., Suvitha A. (2021). Experimental, computational analysis of butein and lanceoletin for natural dye-sensitized solar cells and stabilizing efficiency by iot. *Environment Development and Sustainability*.

[25] Gülcan O., Yiitba S. T., Konukseven E. I. (2021). *Effect of Building Direction on Mechanical Properties of Ti6al4v Parts Produced by Electron Beam Melting*.

